# Paracrine interleukin-8 affects mesenchymal stem cells through the Akt pathway and enhances human umbilical vein endothelial cell proliferation and migration

**DOI:** 10.1042/BSR20210198

**Published:** 2021-05-20

**Authors:** Lulu Wang, Yongtao Li, Xiaodong Zhang, Na Liu, Shiyang Shen, Shizhu Sun, Yang Jiang, Penghui Li, Haifeng Jin, Lei Shen

**Affiliations:** 1 Department of Anatomy, Qiqihar Medical University, Qiqihar, Heilongjiang 161006, P.R. China; 2 Department of Anatomy, Jiamusi University, Jiamusi, Heilongjiang 154007, P.R. China; 3 Grade 2019 of Acupuncture and Massage, Heilongjiang University of Chinese Medicine, Harbin, Heilongjiang 150040, P.R. China; 4 Department of Cell Biology, Qiqihar Medical University, Qiqihar, Heilongjiang 161006, P.R. China

**Keywords:** Bioinformatics, Human bone marrow mesenchymal stem cells, Human umbilical vein endothelial cells, Interleukin-8, Migration, Proliferation

## Abstract

Interleukin-8 (IL-8) promotes cell homing and angiogenesis, but its effects on activating human bone marrow mesenchymal stem cells (BMSCs) and promoting angiogenesis are unclear. We used bioinformatics to predict these processes. *In vitro*, BMSCs were stimulated in a high-glucose (HG) environment with 50 or 100 μg/ml IL-8 was used as the IL-8 group. A total of 5 μmol/l Triciribine was added to the two IL-8 groups as the Akt inhibitor group. Cultured human umbilical vein endothelial cells (HUVECs) were cultured in BMSCs conditioned medium (CM). The changes in proliferation, apoptosis, migration ability and levels of VEGF and IL-6 in HUVECs were observed in each group. Seventy processes and 26 pathways were involved in vascular development, through which IL-8 affected BMSCs. Compared with the HG control group, HUVEC proliferation absorbance value (A value), Gap closure rate, and Transwell cell migration rate in the IL-8 50 and IL-8 100 CM groups were significantly increased (*P*<0.01, *n*=30). However, HUVEC apoptosis was significantly decreased (*P*<0.01, *n*=30). Akt and phospho-Akt (P-Akt) protein contents in lysates of BMSCs treated with IL-8, as well as VEGF and IL-6 protein contents in the supernatant of BMSCs treated with IL-8, were all highly expressed (*P*<0.01, *n*=15). These analyses confirmed that IL-8 promoted the expression of 41 core proteins in BMSCs through the PI3K Akt pathway, which could promote the proliferation and migration of vascular endothelial cells. Therefore, in an HG environment, IL-8 activated the Akt signaling pathway, promoted paracrine mechanisms of BMSCs, and improved the proliferation and migration of HUVECs.

## Introduction

It is estimated that by 2045, the number of people with diabetes worldwide will increase to 693 million, while the current annual global medical expenditure on diabetes is approximately US$ 850 billion [1]. The prevalence of and mortality from diabetes are increasing globally, and have an important impact on global economic development, social stability, financial behavior, and health systems [2].

Hyperglycemic skin ulcer tissues are deficient in cytokines such as interleukin-8 (IL-8), this leads to reduced vascular endothelial cell activity, and a reduced number of peripheral blood vessels, which often promotes issues with the healing of diabetic skin ulcers [3,4]. Homing of host cells to the tissues surrounding a diabetic skin ulcer promotes the repair of ulcers and other injuries [5]. Mesenchymal stem cells (MSCs) can be differentiated into multiple cell types and are widely used in tissue engineering for the repair of injured tissues [6]. Recent studies have found that MSCs effectively promote angiogenesis of ulcerative tissue and accelerate wound healing of diabetic skin ulcers [7,8]. Therefore, the use of MSCs to recruit vascular endothelial cells to home the areas of diabetic skin injury is important for accelerating the repair of diabetic skin ulcers and other complications [9].

Inflammatory factors play important roles in the cell homing process [10,11]. IL-8, which is also known as C–X–C motif chemokine ligand 8 (CXCL-8), is an important member of the CXC chemokine subfamily [12]. It is known that IL-8 is an important factor during the skin wound healing process where it stimulates cell homing and promotes angiogenesis [10,13,14]. However, the reduced cell activity as a result of hyperglycemia, which directly causes a significant reduction in IL-8 and other cytokines in diabetic skin ulcer tissue, inhibits the wound healing of diabetic skin ulcers [15].

Previous studies found that the expression of IL-8 in glioblastoma and melanoma tissue is up-regulated, thereby inducing angiogenesis to promote tumor growth and metastasis [16,17]. Moreover, IL-8 promotes the homing of vascular endothelial cells through the Akt signaling pathway and accelerates the healing of ischemic and hypoxic skin ulcers [18]. Therefore, diabetic vascular disease induces tissue hypoxia. However, under high-glucose (HG) environments, the biological process and molecular mechanisms of IL-8-stimulated MSCs that influence vascular endothelial cells are unclear.

We used bioinformatics to predict the biological process and molecular mechanisms by which IL-8 promotes vascular endothelial cell activation through human bone marrow MSCs (BMSCs). We elucidated the effects of IL-8-stimulated BMSC conditioned medium (CM) on human umbilical vein endothelial cell (HUVEC) proliferation, apoptosis, and migration in an HG environment. We also analyzed the molecular mechanism by which IL-8 acts on BMSCs. These studies will be significant for stimulating host cell homing and promoting the regeneration of diabetic tissue.

## Materials and methods

### Prediction of IL-8 targets and BMSC gene expression profiles

The targets of IL-8 were collected from two databases, namely, the SwissTargetPrediction database (http://www.swisstargetprediction.ch) [19] and the prediction database (http://prediction.charite.de) [20]. The IL-8 targets were determined after removing duplicate values.

The BMSC gene expression profile of the GSE9520 dataset was obtained from the Gene Expression Omnibus (GEO) database (https://www.ncbi.nlm.nih.gov/geo) after setting the adjustment to *P*<0.05. Among these, MSCs were cultured for 2 days, while a separate group of MSCs were cultured for 7 days, and both were used in the present study. The gene expression profile platform was GPL570 [HG-U133_Plus_2], and the GSE9520 series matrix was used with a probe. The common gene expression heat map of IL-8 and BMSCs was prepared using Toolbox for Biologists (TBtools) v1.046 [21].

### Gene ontology and pathway enrichment analysis

The common genes of IL-8 and BMSCs were screened using the Bioinformatics and Evolutionary Genomics online tool (http://bioinformatics.psb.ugent.be/webtools/Venn). The common genes identified by gene ontology (GO) and pathway enrichment analyses were predicted using Metascape Gene Annotation and Analysis Resource (https://metascape.org) [22].

### Screening of protein–protein interactions and core proteins

We determined the expression of common protein interaction between IL-8 and BMSC using the BisoGenet 3.0.0 plug-in of CytoScape3.8 [23]. The core proteins of IL-8 and BMSCs were determined using the CytoNCA2.1.6 plug-in of Cytoscape 3.8, and a degree value with more than two-times the node median was set. In addition, the degree centrality (DC), betweenness centrality (BC), closeness centrality (CC), network centrality (NC), localized average context (LAC) > median of nodes, and IL-8 and BMSC core proteins were identified [24].

### Cell culture

BMSCs were purchased from Cyagen Biosciences (cat. no. HUXMA-01001; Suzhou, Jiangsu, China). HUVECs were purchased from the American Type Culture Collection (cat. no. CRL-4053; Manassas, VA, U.S.A.). Minimum essential medium Eagle-α modification (α-MEM, cat. no. 12571063) and Roswell Park Memorial Institute (RPMI)-1640 (RPMI-1640, cat. no. A4192301; all from Thermo Fisher Scientific, Inc., Waltham, MA, U.S.A.) were used as the basic BMSC medium or the basic HUVEC medium, respectively. Basic medium that contained 300 mmol/l glucose (cat. no. D8270; Sigma, St. Louis, MO, U.S.A.) was established as the cellular HG model environment [25].

### BMSCs experimental groups

Under HG conditions, 4 × 10^6^ BMSCs cultured without any stimulation were defined as the HG-control group. BMSCs treated with 50 or 100 μg/ml human recombinant IL-8 protein (cat. no. 208-IL; R&D, Minneapolis, MN, U.S.A.), and cultured at 37°C and 5% CO_2_ for 12 h, were named as the HG-IL-8_50_ group and HG-IL-8_100_ group, respectively. The cells were cultured with 5 μmol/l Triciribine (Kangchen Biotech, Shanghai, China) at 37°C and 5% CO_2_ for 60 min, washed three times with 0.01 mmol/l phosphate buffered saline (PBS, cat. no. ZLI-9061; Beijing Zhongshan Golden Bridge Technology Co. Ltd., Beijing, China) and then stimulated with 50 or 100 μg/ml of IL-8 protein at 37°C and 5% CO_2_ for 12 h, as the Akt inhibitor group (HG-AI_50_ group and HG-AI_100_ group). BMSCs cultured under normal conditions were used as the normal control group.

### HUVECs grouping

The supernatants of BMSCs were extracted separately from each group and diluted with HUVEC HG medium at a ratio of 1:4 [25]. The diluted supernatants were used as CM, and they were referred to as the HG-control CM group, HG-IL-8 CM group, and HG-Akt inhibitor CM group. Under HG conditions, HUVECs without any stimulation formed the unconditioned medium (NCM) group. Under normal culture conditions, HUVECs without any stimulation were the control group.

### MTT assay

HUVECs were cultured in 96-well plates (Corning, NY, U.S.A.) at 7.5 × 10^3^ cells/well. After discarding the original medium, HUVECs were washed three times with 0.01 mmol/l PBS. New HUVEC HG medium or CM was added according to the HUVEC experimental grouping, and the cells were incubated at 37°C and 5% CO_2_ for 6 h. Subsequently, 0.5% of 3-(4,5-dimethylthiazol-2-yl)-2,5-diphenyltetrazolium bromide (MTT, cat. no. M2128, Sigma, U.S.A.) was added to each well for 4 h at 37°C and 5% CO_2_. Next, 100 μl of dimethylsulfoxide was added to each well (cat. no. 156914; Sigma, U.S.A.), and the samples were shaken for 10 min to fully dissolve the crystals. The absorbance value (A value) of HUVEC proliferation in each group was measured using a Bio-Rad model 550 microplate reader (Hercules, CA, U.S.A.) at 490 nm. Each HUVEC was inoculated in ten wells with three replicates.

### Annexin V-PI apoptosis assay

A total of 2.5 × 10^5^ HUVECs from each group were resuspended in 1.25% Annexin V–fluorescein isothiocyanate (Annexin V–FITC) conjugate solution (cat. no. V13242; Invitrogen, Carlsbad, CA, U.S.A.) and incubated at 4°C for 15 min. The cells were centrifuged for 5 min at 1000 rpm and 4°C, 2% propidium iodide (PI, cat. no. P1304 MP; Invitrogen, Carlsbad, CA, U.S.A.) was added, and the samples were incubated for 3 min. After washing three times with 0.01 mmol/l PBS, the samples were centrifuged at 1000 rpm and 4°C for 5 min, and then resuspended in 0.01 mmol/l PBS. The HUVEC apoptosis rate of each group was determined using a BD FACSAria II flow cytometer (BD Biosciences, Franklin Lakes, NJ, U.S.A.). Each batch of HUVECs was inoculated in ten wells with three replicates.

### Cell scratch experiment

HUVECs were plated in six-well plates (Corning, NY, U.S.A.) at 1 × 10^6^ cells/well. When cells covered the bottom of the well, a central scratch was created by scraping cells away with a p1000 pipette tip, and the stripped cells were washed three times with 0.01 mmol/l PBS. According to the HUVEC experimental grouping, the HUVECs were cultured in HG medium or corresponding CM with 2 mmol/l hydroxyurea (cat. no. H8627; Sigma, U.S.A.) and incubated at 37°C in 5% CO_2_ for 24 h. Then, the cells were rinsed three times with 0.01 mmol/l PBS. The HUVECs were fixed with 4% paraformaldehyde (cat. no. 16005; Sigma, U.S.A.) at room temperature for 2 h and then stained with 1% Crystal Violet (cat. no. C6158; Sigma, U.S.A.). The scratches were recorded with an IX53 inverted fluorescence microscope (Olympus, Tokyo, Japan), and the cell scratch areas at 0 and 24 h were measured using Image-Pro Plus (IPP) 6.0.1 software (Media Cybernetics, Rockville, MD, U.S.A.). The residual rate of the scratch area at 24 h was calculated as follows: (cell scratch area at 24 h/cell scratch area at 0 h) × 100% [26]. Each batch of HUVECs was inoculated in ten wells with three replicates.

### Transwell migration experiment

HUVECs were resuspended in serum-free medium, and 1.0 × 10^4^ cells were loaded into 8.0-μm Transwell cell chambers (Corning, U.S.A.). According to the HUVEC experimental grouping, CM or HG medium (serum-free) were added to the lower chambers. After 12 h of incubation at 37°C and 5% CO_2_, the culture medium was extracted from the Transwell lower chambers in each HUVEC group and centrifuged for 5 min at 800 rpm. The cells were resuspended in 0.01 mmol/l PBS, and the number of cells in the suspension was counted. The non-migrated cells were removed from the Transwell chambers, and the cells were washed three times with 0.01 mmol/l PBS. HUVECs that migrated to the other side of the membrane were fixed with 4% paraformaldehyde (Sigma, U.S.A.) for 2 h and stained with 1% Crystal Violet (Sigma, U.S.A.). Cell migration was observed with an IX53 inverted fluorescence microscope (Olympus, Tokyo, Japan), and the cell migration rate was calculated at 12 h as follows: [(cells in Transwell cell chamber for 12 h + cells in heavy suspension)/1.0 × 10^4^] × 100% [27]. Each batch of HUVECs was inoculated in ten wells with three replicates.

### Enzyme-linked immunosorbent assay

RIPA cell lysis buffer (Beyotime, China) was used to lyse 2.0 × 10^6^ BMSCs in each group. The cells were centrifuged at 12000 rpm at 4°C for 5 min, and the protein was extracted from each group. Total protein content was measured using a BCA protein quantitation kit (Beyotime, China), and 30 μg of each group was used for enzyme-linked immunosorbent assay (ELISA). The BMSC lysates’ contents of Akt and phospho-Akt (P-Akt) in each group were determined by human-Akt (cat. no. DYC1775-5), P-Akt (cat. no. DYC887B-5), and ELISA kit (All R&D, MN, USA). IL-6 and VEGF protein contents in the supernatant of BMSCs in each group were detected via a human IL-6 ELISA kit (cat. no. S6050) and a human VEGF protein and ELISA kit (All R&D, MN, U.S.A.). ELISA was performed according to the manufacturer’s instructions. The protein content of the BMSC lysate or the supernatant in each group was determined from 15 replicates.

### Statistical analysis

The *t* test and variance analyses were performed using Statistical Product and Service Solutions (SPSS) 18.0 for Windows (SPSS, Inc., Chicago, IL, U.S.A.). All of the experimental data have been expressed as means ± SE; all the *P*-values were two-tailed; and *P*<0.05 was considered statistically significant.

## Results

### IL-8 target and BMSC gene expression

The 5129 gene expression profiles of BMSCs were detected from the GSE9520 dataset. Using the STB database and prediction database, a total of 104 IL-8 target genes were predicted. We found 40 common genes between IL-8 and BMSCs, including *EDNRA*, *TACR2*, *CCKAR*, *GHSR*, *SSTR2*, *FNTA*, *SSTR*, *ITGA2B*, *ITGB1*, *NRP1, SSTR5*, *NTSR1*, *NCOR2*, *HDAC1*, *AVPR1A*, *ITGAV*, *CAPN1*, *HDAC2*, *MMP1*, *MMP2*, *PPARG*, *ECE1*, *MMP7*, *BACE1*, *EPHX2*, *PTGS2*, *GRB2*, *ITGA3, MEN1*, *CTSC*, *CTSD*, *MLNR*, *CASP1*, *OPRL1*, *PLG*, *ITGA4*, *ITGAL*, *ITGB2*, *ICAM1*, and *ITGB3* (Figure 1).

**Figure 1:** Gene expression of IL-8 and BMSC (**A**) Venn analysis of IL-8 and BMSC gene expression. (**B**) Common gene expression profile heat map of IL-8 and BMSCs as detected by the GSE9520 dataset. The Pearson correlation distance metric and the average linkage clustering algorithm were used.

### GO analysis

Among the 40 common genes between IL-8 and BMSCs, 53, 495, and 41 were categorized as cellular component (CC), biological process (BP), and molecular function (MF), respectively (*P*<0.05, Figure 2A–C). The 40 common genes were distributed in cell–substrate adherens junctions, extracellular matrices, and other cell sites (Figure 2E). There are approximately 70 major BPs associated with vascular development, promoting vascular endothelial cell proliferation, migration or mesenchymal cell differentiation. These include cell–matrix adhesion, positive regulation of cell motility, blood vessel development, positive regulation of CC movement, angiogenesis, blood vessel morphogenesis, blood circulation, positive regulation of cell death, endothelial cell migration, endothelial cell proliferation, positive regulation of vasculature development, regulation of angiogenesis, regulation of vasculature development, vascular endothelial cell proliferation, positive regulation of sprouting angiogenesis, regulation of nitric oxide biosynthetic process, blood vessel endothelial cell migration, sprouting angiogenesis, vascular endothelial growth factor receptor signaling pathway, cell migration involved in sprouting angiogenesis, positive regulation of endothelial cell migration, regulation of sprouting angiogenesis, and mesenchymal cell differentiation. A total of 37 genes were identified, of which 17 genes occurred more frequently than the median, including *PTGS2*, *NRP1*, *ITGB2*, *ITGB1*, *ICAM1*, *ITGB3*, *PPARG*, *ITGA4*, *GHSR*, *ITGAV*, *ITGA3*, *EDNRA*, *AVPR1A*, *ECE1*, *PLG*, *GRB2*, and *MEN1* (Figure 2D). The molecular functions related to vascular development included G protein-coupled peptide receptor activity, C–X3–C chemokine binding, extracellular matrix binding, cell adhesion molecule binding, cytokine binding, and growth factor binding. A total of 38 genes were identified, of which 17 genes occurred more frequently than the median, including *ITGAV*, *ITGB1*, *ITGB3*, *CTSC, ECE1*, *AVPR1A*, *MMP1*, *MMP2*, *MMP7*, *PLG*, *PPARG*, *SSTR2*, *CASP1*, *HDAC1*, *ITGA4*, *SSTR3*, and *SSTR5* (Figure 2F).

**Figure 2:** GO analysis of the genes common to IL-8 and BMSCs (**A–C**) Enrichment analysis histogram of the BP, CC, and MF of the genes common to IL-8 and BMSCs. The y-axis indicates different GO terms and the x-axis indicates the enrichment score in each category. (**D–F**) Chordal graph of IL-8 and BMSCs common genes with BP, CC, and MF.

### Pathway analysis

Pathways with 40 genes common to IL-8 and BMSCs had 47 items (*P*<0.05), as shown in Figure 3A. There were 26 pathways related to neovascularization, including the PI3K Akt signaling pathway, pathways in cancer, cell adhesion molecule pathways, ECM–receptor interaction pathways, focal adhesion pathway, cAMP signaling pathway, calcium signaling pathway, Rap1 signaling pathway, etc. A total of 37 genes were identified, including 18 genes with frequencies above the median: *ITGB1*, *ITGB3*, *ITGAV*, *GRB*2, *ITGA2B*, *ITGB2*, *HDAC1*, *ITGA4*, *HDAC2*, *ICAM1*, *ITGA3*, *ITGAL*, *PTGS2*, *MMP2*, *PPARG*, *EDNRA*, *MMP1*, and *PLG* (Figure 3B).

**Figure 3:** Common genes pathway analysis of IL-8 and BMSCs (**A**) Pathway enrichment analysis bubble chart of genes common to IL-8 and BMSC. The y-axis indicates different pathway terms and the x-axis indicates the enrichment score in each category. (**B**) Chordal graph of genes common to IL-8 and BMSCs with pathways.

### Protein interaction of IL-8 and BMSC common genes

There were 2483 nodes and 55875 lines in the protein interaction network of common genes between IL-8 and BMSCs (Figure 4A). The main core proteins included RPL5, L7A, S2, S6, S8, L14, L4, L6, L11, L19, L18, S3A, S4X, S15A, S5, S24, L23, S19, SA, L23A, LP0, S3, S7, L8, L24, S20, S18, S11, S28, L36, S15, F3, CL, HNRNPM, ILF2, PABPC1, EEF2, RACK1, HNRNPK, PARP1, and HNRNPR (Figure 4B).

**Figure 4:** Network construction of IL-8 and BMSC gene protein interaction, and screening of core proteins (**A**) The protein interaction network of IL-8 and BMSC genes. (**B**) Strategy diagram of IL-8 and BMSC core protein screening. The node area or font size is positively correlated with the wiring of the node. DC, BC, Closeness centrality (CC), NC, LAC.

### The effect of CM in each group on HUVEC proliferation

To determine the effect of each BMSC-CM on HUVEC growth under HG conditions, we performed an MTT assay to examine HUVEC proliferation. Compared with the HG-NCM group and HG-control CM group, the A values of HUVEC proliferation increased gradually in the HG-IL-8_50_ CM and HG-IL-8_100_ CM groups (*P*<0.05, Figure 5A). Moreover, the A value of HUVEC proliferation in the HG-IL-8_100_ CM group was 1.465-fold higher than that of the HG-IL-8_50_ CM group (*P*<0.01, Figure 5A). By comparison, the A values of HUVEC proliferation in the HG-AI_50_ CM and HG-AI_100_ CM groups were 0.532- and 0.310-fold that of the HG-IL-8_50_ CM and HG-IL-8_100_ CM groups, respectively (all *P*<0.01, Figure 5A).

**Figure 5:** In an HG environment, IL-8 stimulated BMSC-CM increased HUVEC proliferation and migration, as well as inhibited HUVEC apoptosis (**A**) MTT assay was used to detect the proliferation of HUVECs, *P<0.05, ^#^*P*<0.01, ^△^*P*<0.01 (*n*=30). (**B**) The comparison of HUVEC apoptosis rate in each group, *P<0.01, ^#^*P*<0.01, ^△^*P*<0.01 (*n*=30). (**C**) HUVEC apoptosis was detected by Annexin V-PI flow cytometry. (**D**) Scratch closure rate of HUVECs in each group. *P<0.05, ^#^*P*<0.05, ^△^*P*<0.05 (*n*=30). (**E**) The migration rate of HUVECs in each group. *P<0.01, ^#^*P*<0.01, ^△^*P*<0.01 (*n*=30). (**F**) Representative images of wound healing in each treatment group after 24 h of culture. Scale bar = 100 µm. The black line represents the scratch area at 0 h. (**G**) Representative images of HUVEC migration in each treatment group after 24 h of culture. Scale bar = 100 µm.

### The effect of CM in each group on HUVEC apoptosis

To explore the effects of CM on HUVEC apoptosis, an Annexin V–PI cell apoptosis assay was used. We found that the apoptosis rate of HUVECs in the HG-IL-8_50_ CM group and HG-IL-8_100_ CM group decreased gradually compared with those in the HG-NCM group and HG-control CM group (*P*<0.01, Figure 5B,C). Meanwhile, the apoptosis rate of HUVECs in the HG-IL-8_100_ CM group was 0.395-fold that of the HG-IL-8_50_ CM group (*P*<0.01, Figure 5B,C). In contrast, the apoptosis rates of HUVECs in the HG-AI_50_ CM and HG-AI_100_ CM groups were 1.372- and 1.135-fold higher than those of the HG-IL-8_50_ CM group and HG-IL-8_100_ CM group, respectively (all *P*<0.01, Figure 5B,C). These results suggest that in an HG environment, the BMSC-CM, stimulated by IL-8, contained cytokines that inhibited HUVEC apoptosis.

### The effect of CM in each group on HUVEC migration

To determine the effects of IL-8-stimulated BMSC-CM on HUVEC movement, we performed HUVEC scratch experiments and Transwell cell migration experiments. The cell scratch experiment revealed that the closure rate of the HUVEC scratch area in the HG-IL-8_50_ CM and HG-IL-8_100_ CM groups increased gradually compared with the HG-NCM and HG-control CM groups (*P*<0.05, Figure 5D,F). However, compared with the HG-IL-8_50_ CM and HG-IL-8_100_ CM groups, the closure rates of HUVEC scratch areas in the HG-AI_50_CM and HG-AI_100_ CM groups decreased by 47.162 and 38.014%, respectively (all *P*<0.05, Figure 5D,F).

Next, in the Transwell cell migration experiment, we found that when compared with the HG-NCM and the HG-control CM groups, the HUVEC migration rates in the HG-IL-8_50_ CM and HG-IL-8_100_ CM groups gradually increased (*P*<0.01, Figure 5E,G). Additionally, when compared with the HG-IL-8_50_ CM group, the HUVEC migration rate in the HG-IL-8_100_ CM group increased by 29.021% (*P*<0.01). In contrast, compared with the HG-IL-8_50_ CM and HG-IL-8_100_ CM groups, the HUVEC migration rates in the HG-AI_50_ CM and HG-AI_100_ CM groups have decreased by 41.204 and 30.994%, respectively (all *P*<0.01, Figure 5E,G). These results suggest that IL-8 may regulate cytokine expression to promote the migration of HUVECs through the Akt signaling pathway.

### VEGF and IL-6 protein expression in BMSCs in each group

To better reveal the effect of IL-8-stimulated BMSC-CM on HUVEC activity, the supernatant of BMSCs in each group was analyzed using ELISA. The results showed that, compared with the HG control group, the protein expression of VEGF protein or IL-6 protein in the HG-IL-8_50_ and HG-IL-8_100_ groups was gradually increased (*P*<0.01, Figure 6A,B). In addition, VEGF protein expression in the HG-AI_50_ and HG-AI_100_ groups was 0.628- and 0.521-fold in the HG-IL-8_50_ and HG-8_100_ groups, respectively (*P*<0.01, Figure 6A). The protein expression of IL-6 protein in the HG-AI_50_ and HG-AI_100_ groups was 0.577- and 0.558-fold in the HG-IL-8_50_ and HG-IL-8_100_ groups, respectively (*P*<0.01, Figure 6B). We detected the expression of Akt protein in lysates and phosphorylated Akt protein by ELISA. We found that, compared with the HG control group, the expression of Akt protein and phosphorylated Akt protein gradually increased in the HG-IL-8_50_ group and the HG-IL-8_100_ group (*P*<0.01, Figure 6C,D). The expression levels of Akt protein in the HG-AI_50_ and HG-AI_100_ groups were 0.511- and 0.714-fold higher than those in the HG-IL-8_50_ and HG-8_100_ groups, respectively (*P*<0.01, Figure 6C). The expression levels of phosphorylated Akt protein in the HG-AI_50_ and HG-AI_100_ groups were only 0.553- and 0.676-fold higher than those in the HG-IL-8_50_ and HG-IL-8_100_ groups (*P*<0.01, Figure 6D). These results suggest that IL-8 may promote the paracrine secretion of VEGF protein or IL-6 protein by activating the Akt signaling pathway.

**Figure 6:** IL-8 promoted Akt protein expression in HG-IL-8_50_ and HG-IL-8_100_ groups, as well as up-regulation of VEGF and IL-6 protein (**A**) The content of VEGF protein in the supernatant of BMSCs was determined by ELISA. *P<0.01, ^#^*P*<0.05, ^△^*P*<0.01 (*n*=15). (**B**) The content of IL-6 protein in each BMSC supernatant was determined by ELISA. *P<0.01, ^#^*P*<0.01, ^△^*P*<0.01 (*n*=15). (**C**) The content of Akt protein in BMSC lysates was determined by ELISA. *P<0.01, ^#^*P*<0.01, ^△^*P*<0.01 (*n*=15). (**D**) The content of P-Akt protein in each BMSC cohort was determined by ELISA. *P<0.01, ^#^*P*<0.01, ^△^*P*<0.01 (*n*=15).

## Discussion

Diabetic angiopathy and cellular dysfunction are the main causes of delayed healing of diabetic skin ulcers [28]. MSCs have been widely applied in the treatment of skin wounds, heart disease, central nervous system injuries, and other diseases [6]. The multiple cytokines secreted by MSCs can promote angiogenesis and have beneficial effects on the treatment of vascular-deficient diseases. Therefore, MSC transplantation is an effective way to treat diabetic complications [29,30]. However, diabetic patients with persistent hyperglycemia have inhibited MSCs, cell viability issues, and delayed tissue recovery. Recruitment of the patient’s own bone marrow MSCs, vascular endothelial cells, and other cells to the area of the skin ulcer may improve the repair of damaged tissue and reduce the risk of tumorigenicity of allografted MSCs.

Recent studies have demonstrated that chemokines are a family of proteins that recruit cells for homing and regulating cell function, and they play an important role in tumorigenesis, tissue regeneration, and repair [11]. It has been reported that in tumors larger than 2 mm, tumor tissue needs local vessels to provide higher levels of oxygen and nutrition [31]. However, in cervical cancer tissue with a diameter of less than 2 mm, blood vessels are not abundant, resulting in a local hypoxic environment. Moving on from this, persistent hypoxia can stimulate HeLa cells to express high IL-8 in cervical cancer, inhibit the apoptosis of HeLa cells, and promote angiogenesis in tumor tissues [32]. These studies indicate that IL-8 has antihypoxic, recruitment of cell homing, and angiogenesis-promoting functions. Our previous studies also found that IL-8 promotes vascular endothelial cell homing in tissues and accelerates the healing of ischemic and hypoxic skin ulcers [18]. The diabetic hyperglycemic environment already exhibits pathological changes, such as small vessel injury and blocked vessels, resulting in local hypoxia. Therefore, we believe that IL-8 also has an important role in the hypoxic environment induced by diabetes mellitus.

In the process of skin wound healing, IL-8 mobilizes the MSCs of adipose tissue and blood vessels to the wound site by combining the CXCR1/2 receptors on the surface of MSCs [33]; this process is important for the promotion of angiogenesis and the repair of skin wounds. However, cellular activity of the local tissue is reduced at the site of diabetic angiopathy, and low secretion levels of IL-8 and other proteins seriously inhibits cell homing and delays wound healing [34]. A high concentration of chemokines recruits host cells for homing [11], and IL-8 exerts a complex influence on MSCs and vascular endothelial cells in the human body. However, under an HG environment, the effects and mechanisms of IL-8 on vascular endothelial cells via the stimulation of MSCs are unclear.

Bioinformatics technology found that IL-8 shares 40 genes with BMSCs, indicating that IL-8 can exert biological effects through BMSCs. *PTGS2*, *NRP1*, *ITGB2*, *ITGB1*, *ICAM1*, *ITGB3*, *PPARG*, *ITGA4*, *GHSR*, *ITGAV*, *ITGA3*, *EDNRA*, AVPR1A, ECE1, *PLG*, *GRB2*, and *MEN1* genes were clearly related to vascular endothelial cell proliferation, endothelial cell migration, positive regulation of vasculature development, and positive regulation of sprouting angiogenesis. These findings show that IL-8 promoted the differentiation of BMSCs and the biological process of the vascular endothelial growth factor receptor signaling pathway.

Our current experiments found that IL-8-stimulated BMSC-CM promoted scratch closure rate and migration rate in HUVECs. With increasing IL-8 concentration, the cell migration and A values of cell proliferation in the CM groups of BMSCs stimulated by IL-8 increased gradually, and the apoptosis rates showed a downward trend; all results exhibited a dose-dependent effect. This may be because IL-8 activates the Akt signaling pathway in BMSCs and then activates the expression of VEGF and IL-6 genes downstream of the Akt signaling pathway to promote the paracrine secretion of VEGF and IL-6 proteins in BMSCs [35,36]. VEGF and IL-6 play an important role in promoting cell activity [37,38]. Bioinformatics also predicted that IL-8 could play a role in the vascular endothelial growth factor receptor signaling pathway of MSCs.

There were 26 pathways related to the expression of IL-8 in BMSCs; pathways related to the proliferation of neovascularized vascular endothelial cells were mostly as follows: the PI3K-Akt signaling pathway, pathways in cancer, and cell adhesion molecules and ECM–receptor interaction pathways. The Akt signaling pathway is a complex signaling network that is known to be involved in maintaining cell homeostasis and is closely related to cell proliferation, cell differentiation, cell motility, and angiogenesis [39]. Moreover, the Akt signaling pathway also plays a key role in the growth and metastasis of small cell lung cancer, colon cancer, and breast cancer [40,41].

Stromal cell-derived factor 1α (SDF-1α) is an important chemokine that is also known as CXCL-12 and belongs to the same family as IL-8 [42,43]. It can activate Akt signaling pathways and promote angiogenesis [44]. Furthermore, it reduces apoptosis of endothelial progenitor cells by activating PI3K/Akt/eNOS [45]. IL-8 is highly expressed in tumor tissues such as gastric cancer and colon cancer and can also initiate the Akt signaling pathway or Hedgehog signaling pathway to improve the growth and metastatic conditions of tumor tissue [46–48]. Yang et al. evaluated the recruitment of BMSCs and the effect of IL-8 in bone regeneration. The results show that IL-8 triggers BMSC migration *in vitro* through the CXCR2-mediated PI3K/Akt signaling pathway. Moreover, *in vivo*, IL-8 induces BMSC cartilage differentiation through the CXCR2-mediated PI3k/Akt signaling pathway [49]. SDF-1/CXCR4 stimulates the expression of IL-8 in pharyngeal squamous cell carcinoma cells through the Akt pathway and promotes tumor angiogenesis [44]. It is important to understand that IL-8 promotes the proliferation or migration of vascular endothelial cells.

In view of the effect of IL-8 on MSC biological process characteristics, when combined with the Akt pathway, IL-8 plays an important role in tumor tissue and embryonic angiogenesis. *In vitro* experiments showed that IL-8 can activate the Akt signaling pathway, promote the secretion of VEGF and IL-6 proteins in addition to BMSCs, and activate vascular endothelial cells.

The current results showed that, in an HG environment, IL-8 plays an important role in enhancing the secretion of BMSCs and promoting the proliferation, movement, and angiogenesis of vascular endothelial cells. However, other molecular mechanisms and biological processes of IL-8 in BMSCs require further study. These results suggest a new protocol for the mobilization of MSCs to participate in angiogenesis.

## Conclusions

Bioinformatics analysis confirmed that IL-8 promoted BMSCs expression of 41 core proteins, including RPL5, L7A, and S2, through 26 pathways including PI3K-Akt, cell adhesion molecule pathways, and ECM–receptor interaction pathways. There are approximately 70 BPs related to vascular development, such as cell matrix adhesion, blood vessel endothelial cell migration, endothelial cell promotion, and spring angiogenesis. In an HG environment, IL-8 activates the Akt signaling pathway, promotes the paracrine mechanism of BMSCs, and improves the proliferation and migration of HUVECs.

## Data Availability

The data used to support the findings of the present study are included within the article.

## Abbreviations

A value: absorbance value
BMSC: human bone marrow mesenchymal stem cell
BP: biological process
CM: conditioned medium
CXCL-8: C–X–C motif chemokine ligand 8
ELISA: enzyme-linked immunosorbent assay
GO: gene ontology
HG: high-glucose
HUVEC: human umbilical vein endothelial cell
IL-8: interleukin-8
MF: molecular function
MSC: mesenchymal stem cell
MTT: 3-(4,5-dimethylthiazol-2-yl)-2,5-diphenyltetrazolium bromide
NCM: unconditioned medium
P-Akt: phospho-Akt
PBS: phosphate buffered saline
PPI: protein–protein interaction
